# Diagnostic Value of Magnetic Resonance Diffusion-Weighted Imaging Combined with Routine Scanning in Body Tumors

**DOI:** 10.1155/2022/5799815

**Published:** 2022-07-21

**Authors:** Zhongwei Li, Di Wang, Jinfeng Sun, Guowei Zhang, Jiashou Hu

**Affiliations:** ^1^Department of Radiology, Yantaishan Hospital, Yantai, China; ^2^Diagnostic Radiology Division, 970 Hospital of the PLA JLSF, Yantai, China; ^3^Department of Oncology, 970 Hospital of the PLA JLSF, Yantai, China

## Abstract

The aim of this study was to evaluate the value of whole body magnetic resonance diffusion-weighted imaging (WB-DWI) combined with routine scanning in the diagnosis of body tumors. Sixty-three patients with surgically and pathologically confirmed body tumors admitted to our hospital from October 2019 to October 2021 were scanned by WB-DWI using a 1.5TMR body coil. The images were reconstructed by a three-dimensional maximum intensity projection (3D-MIP) and black-white inversion technique. The lesions detected by WB-DWI were all plain MRI, and 35 cases were enhanced MRI. The number of lesions detected by WB-DWI and WB-DWI combined with routine scanning and the number of cases matching diagnosis were compared. The WB-DWI images of tumor lesions were analyzed, and the apparent diffusion coefficient (ADC) of the lesions was measured, and the ADC value of benign and malignant lesions was compared. There were 236 lesions in 63 patients with clinically confirmed tumors. 46 cases were diagnosed by WB-DWI, the diagnostic coincidence rate was 73.0%, and 207 lesions were detected. Fifty-eight cases were diagnosed by WB-DWI combined with routine scanning, the diagnostic coincidence rate was 92.1%, 236 lesions were detected. There were statistically significant differences in the number of lesions detected and the coincidence rate of tumor diagnosis between the two groups (*P* < 0.05). The average ADC value of malignant tumor ((1.04 ± 0.46) × 10^−3^ mm^2^/s) was lower than that of benign tumor ((2.53 ± 0.43) × 10^−3^ mm^2^/s), and the difference was statistically significant (*P* < 0.05). In conclusion, MR whole-body diffusion weighted imaging is safe, efficient, radiation-free, and highly sensitive, which is of great significance in the differential diagnosis of benign and malignant lesions. WB-DWI combined with MR routine scanning can further improve the detection rate of lesions and the coincidence rate of tumor diagnosis.

## 1. Introduction

Magnetic resonance whole-body diffusion weighted imaging (WB-DWI) is a noninvasive technique to detect the movement of water molecules in living tissues, which is of great value in the detection of primary tumor and metastatic tumor, especially in the differential diagnosis of benign and malignant lesions [1, 2]. This technology has been developed rapidly in recent years. It has high sensitivity, low cost, no radiation, and can detect tumor lesions sensitively, and has been widely applied in clinical practice [3, 4]. This study retrospectively analyzed the data of WB-DWI and MRI routine examination of lesions in 63 patients with body tumor and preliminary discussed the application value of WB-DWI combined with MRI routine examination in the detection of lesions and differential diagnosis of benign and malignant tumors.

## 2. Patients and Methods

### 2.1. Patients

The WB-DWI, plain, and enhanced MRI images of 63 patients with tumor confirmed by surgery and pathology admitted to our hospital from October 2019 to October 2021 were retrospectively analyzed (Table 1). There were 42 males and 21 females, aged from 29 to 78 years, with an average of 54.6 years. All patients underwent plain MRI scan for lesions detected by WB-DWI within 1 week, and 35 patients underwent enhanced MRI scan. Inclusion criteria were as follows: 1. those with a clear diagnosis of tumor and 2. those with no contraindications to MRI. Exclusion criteria were as follows: 1. those who refused to have an MRI and 2. those who had a fear of MRI.

### 2.2. Check Methods

G:E 1.5T superconducting magnetic resonance, with built-in gross coil. WB-DWI scanning parameters: Short T1 flip recovery plane echo dispersion weighted imaging sequence (STIR-EPI-DWI), TR 5100 ms, TE 102.7 ms, TI 180 ms, FOV 40 cm × 40 cm, matrix 96 × 128, NEX6 times, layer thickness 7 mm, layer spacing −1 mm, The B values are 0 s/mm^2^ and 600 s/mm^2^, respectively. Six axial images were collected (from the top of the head to near the knee joint), 60 images were collected at 30 layers in each section, and the scanning time was 4 minutes and 5 seconds. A total of 24 minutes and 30 seconds were required for whole body scanning. All six axial images were selected into the functional software processing system, and 360 axial images were obtained. 180 images with *B* = 600 s/mm^2^ were selected for a 3D-MIP reconstruction and black-white inversion technique.

### 2.3. Image Analysis

Image analysis was performed by two experienced radiologists using a double-blind method. First, the WB-DWI images of each case were analyzed, the number of lesions detected was counted, and the disease diagnosis was made based on the history. Then, WB-DWI was combined with routine scanning for analysis, and the number of detected lesions was counted again, and disease diagnosis was carried out based on medical history and imaging data. For bone lesions, focal lesions were counted by the number of lesions, while diffuse lesions were counted by the unit of bone involved. For the lesions of lymph nodes and other organs, the number of lesions was counted as a unit, the shortest diameter of lymph nodes >1.0 cm could be counted, and the fused masses were counted as a single lesion. Measuring ADC values of tumor lesions, maximum level of selected lesions, avoid the focal necrosis area, hand-painted suitable size round/oval region of interest (ROI) in focal interest areas get the ADC values of corresponding place, within the lesion as far as possible more acquisition ADC values (mainly due to varying degrees at various points within the tumor cells arranged closely, dispersion rate may be different), ADC values were expressed as mean ± standard deviation.

### 2.4. Statistical Analysis

Statistical Product and Service Solutions (SPSS) 20.0 software (IBM, Armonk, NY, USA) was used for statistical analysis of the study data. SPSS 20.0 software offers advanced statistical analysis, a vast library of machine learning algorithms, text analysis, open source extensibility, integration with big data, and seamless deployment into applications. The ADC value was expressed as mean ± standard deviation (x̅ ± *s*), and *t*-test was adopted. *P* < 0.05 was considered statistically significant. *χ*^2^ test was used to compare the degree of consistency between the two diagnostic methods and pathological results.

## 3. Results

Among the 63 tumor patients diagnosed by surgery or biopsy, 236 lesions were detected by WB-DWI combined with routine scanning, and 207 lesions were detected by WB-DWI alone (Table 1), with a sensitivity of 87.7%. There was a statistically significant difference in the number of lesions detected between the two groups (*P* < 0.05). 207 lesions showed high signal intensity on WB-DWI, but the signal intensity was different. 3 nasopharyngeal carcinoma lesions showed a uniform high signal, 8 lung cancer lesions showed homogeneous/slightly uneven mass with slightly high/high signal, and 2 lesions showed an uneven ring high signal. There were 6 primary liver cancers with an uneven slightly high/high signal and 17 liver metastases had a nodular slightly high signal. 4 lesions of pancreatic cancer showed obvious hypersignal mass. Three renal carcinoma lesions showed irregular hypersignal masses, similar to normal renal parenchyma (Figure 1). Three prostate cancer foci were located in the peripheral zone, showing a slightly high signal, which was lower than that in the normal peripheral zone. 17 lymphoma lesions showed an obvious high signal, 33 metastatic lymph nodes presented as nodules/masses with obvious high signal, and 10 nodules with annular high signal. 69 bone metastases showed a pointy and patchy obvious high signal. 20 liver hemangioma lesions showed an obvious high signal and 6 lesions showed a slightly high signal. One lesion of renal eosinophil showed a high signal, slightly higher than that of normal renal parenchyma. One adrenal myelolipoma showed slightly higher signal (Figure 2). One lesion of ovarian teratoma showed high and low mixed signals. Three uterine fibroids showed slightly higher signal intensity. The above 207 lesions showed a corresponding degree of low signal on the black-white inversion image, and the average ADC values of various tumors are shown in Table 2.

The diagnostic comparison of 63 patients with WB-DWI and WB-DWI combined with MRI routine scanning is shown in Table 3, and there was statistically significant difference in the coincidence rate of tumor diagnosis between the two groups (*P* < 0.05). The average ADC values of benign and malignant tumors in body parts are compared in Table 4, and the difference between them was statistically significant (*P* < 0.05).

## 4. Discussion

### 4.1. Magnetic Resonance Whole Body Diffusion-Weighted Imaging Technique

Magnetic resonance diffusion weighted imaging (DWI) is a noninvasive technology for detecting the motion of water molecules in living tissues, which shows the Brownian motion of water molecules. It is the only method that can measure and image the dispersion of water molecules in living tissues. WB-DWI is a combination of DWI, echo planar imaging (EPI), and short time inversion recovery (STIR) fat suppression technology to complete a wide range of scans under the condition of free breathing. The images are reconstructed by 3D-MIP and processed by black-white inversion. Higher gradient field strengths and gradient switching rates increase imaging speed, minimize echo time (TE), and improve image signal-to-noise ratios. The single excitation EPI technology is used to collect all the K-space data at one time, and an image can be completed in sub-second time, which minimizes the error caused by motion and reduces motion artifacts, so as to achieve high resolution and high signal-to-noise ratio image acquisition under free breathing. The STIR technology can effectively suppress fat, reduce background noise, increase image contrast, improve reconstructed image quality, and clearly display normal tissues and lesions [5].

### 4.2. Clinical Significance of the ADC Value

The apparent diffusion coefficient (ADC) value is usually used to replace the true diffusion coefficient D. In diffusion weighted imaging, molecular dispersion is also affected by factors such as blood flow, cerebrospinal fluid flow, macroscopic movement, cell membrane, etc. The ADC value integrates the above factors and can reflect the characteristics of the overall tissue structure [6]. ADC value is also related to the *b* value of the diffusion weighted imaging coefficient. As the B value increases, the ADC value is closer to the *D* value, but as the *B* value increases, the signal-to-noise ratio of the DWI image gradually decreases and the magnetic sensitivity artefacts increase. Low et al. [7] believed that when *B* = 400–600 s/mm^2^, high-quality images could be obtained and anatomical structures could be clearly displayed. The solid part of malignant tumor cells grew actively and arranged closely. The biofilm structure clearly limits the diffusion of water molecules, the ADC value decreases, and DWI shows a high signal. In contrast, benign tumors have low cell density, relatively large ADC values and relatively low signal on DWI. Cytotoxic edema or the increase in cellular volume restricts the Brownian motion of water molecules. Some benign lesions can also cause diffuse weakening, while vasogenic edema can cause diffuse enhancement, which leads to the intersection of ADC values of benign and malignant lesions, especially in inflammatory lymph nodes, metastatic lymph nodes, and lymphoma. In this study, the average ADC value of renal cancer was higher than that of benign tumor. Therefore, a comprehensive analysis of imaging data such as WB-DWI and MRI routine examination was required for differential diagnosis of benign and malignant lesions.

### 4.3. Clinical Application of Whole-Body Diffusion-Weighted Magnetic Resonance Imaging Combined with Routine Scanning

MR whole body diffusion-weighted imaging can better display thyroid, spleen, kidney, bladder, intervertebral disc, prostate, uterus and lymph nodes, and other tissue structures, with a large scanning coverage, short scanning time, no radiation, no contrast agent, high sensitivity, and other characteristics. As two imaging methods for whole-body tumor screening, WB-DWI and PET-CT have the advantages of noninvasiveness, no radiation, low cost, and sensitive detection of tumor lesions [3, 4, 8] and are increasingly favored by clinicians and patients. WB-DWI has an important clinical application value in detecting the primary tumor, local lymph node, and distant metastasis of malignant tumor. Compared with PET-CT, each of them has advantages and complement each other [6–9]. Ono et al. [10] compared DWI and PET in 25 patients with colorectal cancer and found that DWI was superior to PET in the detection of lymph node metastasis. The study of Usuda et al. [11, 12] showed that in the qualitative diagnosis of hilar and mediastinal lymph nodes, DWI based on the quantitative analysis of suspicious lymph node ADC can effectively distinguish inflammatory and cancerous lymph nodes, which is of great significance for tumor N staging. WB-DWI can effectively evaluate the tumor efficacy. The comparison of WB-DWI images of 29 patients with malignant tumor before and after clinical treatment showed that 75% of the lesions were reduced in volume and ADC value significantly increased after treatment, and lymph node metastasis and distant metastasis were found in 13 of them. The article was a single-center study and there may be some bias in the selection of patients. Therefore, a multicentral, randomized, and double-blind study was needed to further confirm the findings of this study.

In conclusion, MR whole-body diffusion-weighted imaging, as a new type of examination method, has the advantages of rapidity, noninvasiveness, nonradiation, and sensitivity to the pathological changes of tumors. By analyzing ADC values combined with conventional MRI scans, we can preliminarily determine whether the tumor is benign or malignant. This technology has unique advantages and application value in tumor diagnosis and prognosis prediction.

## Figures and Tables

**Figure 1:** Kidney cancer. (a) WB-DWI image showed a significant low signal shadow in the right kidney with a range of 5.3 cm × 4.4 cm. (b) T1WI showed the lesion with low signal. (c) Lipid-suppressed T2WI showed hyperintense lesions with well-defined edges and areas of liquefaction necrosis. (d) Gd-DTPA dynamic enhanced scanning in arterial phase, the solid part of the lesion was significantly enhanced with clear boundary. (e) Lesion enhancement decreased during the coronal equilibrium phase.

**Figure 2:** Adrenal myelolipoma. (a) WB-DWI image showed patchy low signal shadow in the left adrenal area. (b) Fat suppression T2WI showed a 2.2 cm × 2.9 cm oval lesion in the left adrenal gland, with clear edge, slightly high signal, and uneven signal. (c) Positive phase diagram of T1WI double echo sequence showed isosignal of the lesion. (d) Inverse phase diagram of double echo sequence showed that the signal of the lesion is significantly reduced.

**Table 1:** Type, metastasis and number of tumors.

Tumor type combined metastatic site	The number of cases
Nasopharyngeal carcinoma	3
*with skull base bone metastasis*	1
Lung cancer	13
*with mediastinal/cervical lymph node metastasis*	8
*with bone metastases*	2
*with multiple liver metastases*	1
Hepatocellular carcinoma	6
*with multiple liver and bone metastases*	2
Pancreatic cancer	4
*with retroperitoneal lymph node metastasis*	2
Kidney cancer	5
*with bone metastases*	1
*with retroperitoneal lymph node me*tastasis	2
Prostate cancer	4
*with bone metastases*	1
Lymphoma	5
Hepatic hemangioma	15
Renal eosinophil tumor	1
Adrenal myelolipoma	1
Ovarian teratoma	1
Uterine fibroids	5

**Table 2:** Comparison of the number of lesions detected by WB-DWI and WB-DWI combined with routine scanning and the ADC value of tumor lesions (×10^−3^ mm^2^/s) (*b* = 600 s/mm^2^).

Tumor type	The number of lesions detected by WB-DWI combined with routine scan	The number of lesions detected by WB-DWI	The average ADC values
Nasopharyngeal carcinoma	3	3	0.92 ± 0.41
Lung cancer	13	10	1.38 ± 0.48
Hepatocellular carcinoma	6	6	1.21 ± 0.29
Liver metastases	28	17	1.19 ± 0.52
Pancreatic cancer	4	4	1.48 ± 0.65
Kidney cancer	5	3	2.42 ± 0.33
Prostate cancer	4	3	1.26 ± 0.57
Lymphoma	17	17	0.97 ± 0.69
Metastatic lymph node	43	43	0.93 ± 0.31
Bone metastases	69	69	0.85 ± 0.53
Hepatic hemangioma	34	26	2.73 ± 0.41
Renal eosinophil tumor	1	1	2.63
Adrenal myelolipoma	1	1	2.45
Ovarian teratoma	1	1	1.59
Uterine fibroids	7	3	2.01 ± 0.35

**Table 3:** Diagnostic comparison of 63 patients with WB-DWI and WB-DWI combined with MRI routine scanning.

Diagnostic methods	Benign tumor	Malignant tumor	Tumor diagnosis coincidence rate
WB-DWI scanning	16	30	73.0%
WB-DWI combined with MRI routine scanning	22	36	92.1%
*χ * ^2^ value			0.109
*P* value			0.048

**Table 4:** Comparison of ADC values of benign and malignant tumors in body (×10^−3^ mm^2^/s).

Tumor types	Number of lesions	Maximum average ADC value	Minimum average ADC value	Average ADC values
Benign tumor	32	2.67 ± 0.49	1.59 ± 0.38	2.53 ± 0.43
Malignant tumor	175	2.46 ± 0.38	0.87 ± 0.46	1.04 ± 0.46
*t* value		2.74	8.34	17.01
*P* value		0.01	＜0.001	＜0.001

## Data Availability

The datasets used and analyzed during the current study are available from the corresponding author on reasonable request.
